The article "Analysis of the Diagnosis Model of Peripheral Non-Small-Cell Lung Cancer under Computed Tomography Images" was retracted in 2023. Reasons: signs of a paper mill; suspected computer-generated content; unreliable results or conclusions; lack of ethics approval or compliance.

# Analysis of the Diagnosis Model of Peripheral Non-Small-Cell Lung Cancer under Computed Tomography Images

**DOI:** 10.1155/2022/3107965

**Published:** 2022-02-18

**Authors:** Zhonghai Xie, Huaizhong Zhang

**Affiliations:** ^1^Huzhou Central Hospital, Huzhou 313000, Zhejiang, China; ^2^Lishui City People's Hospital, Lishui 323000, Zhejiang, China

## Abstract

This study aimed to explore the effect of deep learning models on lung CT image lung parenchymal segmentation (LPS) and the application value of CT image texture features in the diagnosis of peripheral non-small-cell lung cancer (NSCLC). Data of peripheral lung cancer (PLC) patients was collected retrospectively and was divided into peripheral SCLC group and peripheral NSCLC group according to the pathological examination results, ResNet50 model and feature pyramid network (FPN) algorithm were undertaken to improve the Mask-RCNN model, and after the MaZda software extracted the texture features of the CT images of PLC patients, the Fisher coefficient was used to reduce the dimensionality, and the texture features of the CT images were analyzed and compared. The results showed that the average Dice coefficients of the 2D CH algorithm, Faster-RCNN, Mask-RCNN, and the algorithm proposed in the validation set were 0.882, 0.953, 0.961, and 0.986, respectively. The accuracy rates were 88.3%, 93.5%, 94.4%, and 97.2%. The average segmentation speeds in lung CT images were 0.289 s/sheet, 0.115 s/sheet, 0.108 s/sheet, and 0.089 s/sheet. The improved deep learning model showed higher accuracy, better robustness, and faster speed than other algorithms in the LPS of CT images. In summary, deep learning can achieve the LPS of CT images and show excellent segmentation efficiency. The texture parameters of GLCM in CT images have excellent differential diagnosis performance for NSCLC and SCLC and potential clinical application value.

## 1. Introduction

Due to the continuous expansion of the number of smokers and the increasingly serious environmental pollution, the incidence of lung cancer in recent years has shown an increasing trend year by year. Clinically, lung cancer is mainly divided into SCLC and NSCLC. NSCLC can be classified into adenocarcinoma, squamous cell carcinoma, adenosquamous carcinoma, and large cell lung cancer [1, 2]. According to the difference of the location of lung cancer lesions, it can be classified into the central type and peripheral type. PLC is the most common type of adenocarcinoma. Peripheral SCLC is relatively rare in clinical practice. Because its pathogenesis is mainly the downward growth of the bronchial mucosa and the infiltration of connective tissue adjacent to the bronchus, the early clinical symptoms are not obvious [3]. The lesion location of peripheral NSCLC is mainly below the segmental bronchus. It is difficult for fiberoptic bronchoscopy to reach the lesion location, and it is difficult to perform puncture cytology for lesions far from the chest wall. Therefore, other methods have to be found for the differential diagnosis of the peripheral NSCLC [4, 5].

Chest CT image is one of the most routine and important diagnostic methods for lung cancer. It can early and clearly find the size, shape, and extent of the patient's lung lesions, so it is often used for the detection, identification, staging, and treatment of lung cancer [6]. With the continuous development of CT technology, the current scanned images of each layer thickness can reach 500. As the method of manual reading and manual segmentation of the location of the lesion increases the workload of the doctor, it also shows some limitations such as low efficiency, subjective misdiagnosis, and missed diagnosis [7]. There have been many studies using machine learning and deep learning technologies to achieve computer-aided diagnosis (CAD) of diseases to make full use of the effective information in CT images and improve the clinical diagnosis rate of diseases [8]. Convolutional Neural Networks (CNNs) are often used in medicine to learn original images and are widely used in image segmentation, image classification, and target image positioning. Mask R-CNN network is used to reconstruct the CT image and build a deep learning network model to enhance the ability of image reconstruction. Some scholars also use artificial intelligence recognition capabilities to read CT images and improve the relevant parameters of the Mask R-CNN model. The network environment constructed by measuring the sharp angle comparison has greatly promoted the reconstruction of the model and improved the intelligent model for auxiliary diagnosis. Deep learning CNN almost has the same value in bone maturity evaluation and manual evaluation. However, the descriptions of machine learning algorithms used for lung lesion feature recognition are all designed by human experience. In the face of complex lesions, it is not able to distinguish features well, and it is difficult to improve the detection accuracy of lung lesions. However, the deep learning model has excellent generalization capabilities. It uses network design to capture the high-dimensional features and obtain a more reliable segmentation model. Therefore, it has been widely used in CAD systems [9].

An algorithm for LPS of lung CT images was proposed based on a deep learning model to improve the efficiency of clinical diagnosis of peripheral NSCLC and peripheral SCLC, and then, it was trained and verified. The CT images of patients with clinical peripheral NSCLC and peripheral SCLC were undertaken as objects, and texture features were extracted based on the images after LPS, so as to compare and analyze the differences in the texture features of CT images of patients. In this way, the quantitative information used in the differential diagnosis of peripheral NSCLC in CT images was excavated to provide a basis for follow-up clinical precision treatment.

## 2. Basic Theories

### 2.1. Basic Theories for Auxiliary Diagnosis of Peripheral NSCLC

#### 2.1.1. Imaging Characteristics of Lung CT

The preprocessing of CT images was a key step of using CAD in lung diseases. It could measure the X-ray absorption rate of body tissues and describe the standard quantitative unit of radiation density, which led to a new measurement unit “CT value.” The mathematical expression for calculating the CT value was given as follows:

(1) $$\begin{array}{c} \text{CT}=\frac{\mu_{1}-\mu_{2}}{\mu_{2}}\cdot \alpha . \end{array}$$

In (1), *α* was the graduation factor, *μ*_1_ represented the attenuation coefficient of X-rays penetrating the body tissue, and *μ*_2_ referred to the X-ray attenuation coefficient of the standard level.

If the attenuation coefficient of water was undertaken as the standard, the CT value at the center at this time could be set to 0 Hu. Then, the maximum CT value of bone was 1000 Hu, and the CT value of lung tissue was in the range of −500∼900 Hu [10]. Since there were 2000 units for the CT value of human tissue, which exceeded the display range of the gray image, so the original CT image was impossible to be analyzed directly by naked eyes. For a specific tissue in the human body, window adjustment technology could be used to display the lesion or marker area as much as possible. The center and width of the window after adjusting the window were the center and range of the CT value of the designated tissue after the linear conversion of the CT value, respectively. Window adjustment could only enable CT images to be accepted by human eyes but could not modify the information of the original CT images, so it was very important in medical CAD systems. The window position of chest CT images was in the range of −600∼700 Hu, and the window width was set to 1000 Hu.

#### 2.1.2. Imaging Findings of Peripheral NSCLC

From a medical perspective, CT signs of lung nodules had specific names and meanings. These signs could help doctors have a better understanding and judgment in the pathological direction, so they were also of great significance for the classification of peripheral NSCLC [11]. The signs of lung nodules firstly showed the “spots” in the chest CT image. If the CT images showed that the patient has lung nodule disease, it was necessary to combine the patient's medical history to understand whether he or she has had cancer, whether he or she has a history of smoking, and whether he or she works in harmful environment, etc. CT image scanning could provide doctors with information about the characteristics of lung nodules, including the shape, size, location, and tissue density of the nodules. In addition, CT images could show small nodules (1∼2 mm in diameter). If the size of the nodules was small enough, it indicated that the possibility of canceration was low. The CT image signs of peripheral NSCLC classification mainly showed the size of the lung nodule, the position of the lung nodule, and the edge and density characteristics of the lung nodule (such as lobes, burrs, Pleural hypertrophy, peripheral emphysema, calcification, satellite foci, cavities, and spinous processes).  Figure 1 shows the CT images of lung nodules A, lung adenocarcinoma B, and lung squamous cell carcinoma C.

### 2.2. Basic Theories of Deep Learning

The continuous development of the digital age had brought about the explosive growth of data, which was referred to as big data. However, it took a long time to use traditional methods to mine effective information in massive data. Therefore, people have tried to use machine learning to process big data. Deep learning was a new field in machine learning, which could make the machine use a nonlinear process to process data through a hierarchical system and then discover the distributed characteristics of the data [12]. In the field of medical imaging, deep learning had also become a very important research tool. It could extract features from images in a self-learning process, so it had certain practical value in medical image segmentation and target detection.

#### 2.2.1. CNN

CNN was an important model for deep learning applied to image processing. It was a training algorithm for deep network models, which could intelligently extract a large number of features and avoid a large amount of calculation and time-consuming training through methods such as local connection and weight sharing. In addition, the model was capable of strong generalization [13].  Figure 2 shows the basic structure of the CNN model, which includes the input layer, convolutional layer, pooling layer, and fully connected layer.

The input layer was used for preprocessing of input image data because the image data inputted to the CNN model belonged to the pixel value matrix, and the range of the pixel code value was determined by the number of coding bits. The color image belonging to the red-green-blue (RGB) channel was inputted into the CNN model as a 3-dimensional vector, which increased the amount of calculation to a certain extent. Therefore, it was necessary to centralize and standardize the input data and input the data that conforms to the normal distribution to the next layer.

The convolutional layer was used for feature processing of input image data. The local perception and weight sharing were to reduce the number of parameters. Since the feature extraction of the convolution kernel was not sufficient, it was necessary to add different convolution kernels to learn different features, and the feature maps generated by each convolution kernel could be regarded as different channels.

The pooling layer was used for the aggregation and statistics of the extracted features of the convolutional layer. The feature size processed by the pooling layer could greatly reduce the calculation amount of the model and prevent the model from overfitting. Pooling operations were divided into maximum pooling and average pooling, which selected the maximum value and average value in the corresponding filter matrix as the outputs, respectively.

The fully connected layer was to learn the label region mapping of the distributed feature vector.

#### 2.2.2. Back Propagation of CNN

The backpropagation of the CNN model referred to the application of chain derivation. For the calculation of CNN's backpropagation algorithm, it was necessary to set the parameters of each layer, including the number of input images and the network layers in the input layer; the size of the convolution kernel, the number of convolution kernel channels, filling size, and step size in the convolutional layer; the filter matrix size and pooling operation mode in the pooling layer; and activation function and the number of nodes in the fully connected layer. In addition, it was necessary to determine the training method, iteration step size, and the threshold for terminating iterations. Finally, the weight value and bias between each network layer in the model were solved, and the specific calculation steps were as follows:

- The weight value *ω* and threshold value *b* of the hidden layer and output layer of the model were initialized and set to random values
- For iter 1 to max:
- For I = 1 to *n* (the maximal number of the inputted images):
- The input *a*_1_ was set to the tensor corresponding to *x*_i_
- For *l* = 2 to *L* − 1 (number of network layer −1), then the following equations could be determined:
- Fully connected layer: *a*_*i*,*l*_=*σ*(*z*_*i*,*l*_)=*σ*(*ω*_*l*_*a*_*i*,*l*−1_+*b*_*l*_)
- Pooling layer: *a*_*i*,*l*_=pool(*a*_*i*,*l*−1_)
- Convolutional layer: *a*_*i*,*l*_=*σ*(*z*_*i*,*l*_)=*σ*(*ω*_*l*_ · *a*_*i*,*l*−1_+*b*_*l*_)
- Then, the outputted layer *L* was defined as *a*_*i*,*L*_=soft max(*z*_*i*,*L*_)=soft max(*ω*_*L*_*a*_*i*,*L*−1_+*b*_*L*_), and the error *ε* of this layer could be calculated further based on the loss function
- For *l* = *L* to 2, then the following equations could be determined:
- Fully connected layer: *ε*_*i*,*l*_=(*ω*_*l*+1_)^*T*^*ε*_*i*,*l*+1_⊙*σ*′(*z*_*i*,*l*_)
- Pooling layer: *ε*_*i*,*l*_=*ε*_*i*,*l*+1_ · rot 180(*ω*_*l*+1_)⊙*σ*′(*z*_*i*,*l*_)
- Convolutional layer: *ε*_*i*,*l*_=up sample(*ε*_*i*,*l*+1_)⊙*σ*′(*z*_*i*,*l*_)
- For *l* = 2 to *L*, the weight of the l-layer network *ω*_l_ and the bias *b*_l_ could be adjusted slightly after the determination:
- Fully connected layer: *ω*_*l*_=*ω*_*l*_ − *λ*∑_*i*=1_^*n*^*ε*_*i*,*l*_(*a*_*i*,*l*−1_)^*T*^ and *b*_*l*_=*b*_*l*_ − *λ*∑_*i*=1_^*n*^*ε*_*i*,*l*_
- Convolutional layer: *ω*_*l*_=*ω*_*l*_ − *λ*∑_*i*=1_^*n*^*ε*_*i*,*l*_ · rot 180(*a*_*i*,*l*−1_) and *b*_*l*_=*b*_*l*_ − *λ*∑_*i*=1_^*n*^∑_*u*,*v*_(*ε*_*i*,*l*_)_*u*,*v*_
- If both the weight value and the bias were less than the termination iteration threshold, the loop was completed
-  The weight value *ω* and threshold value *b* of the hidden layer and output layer were outputted

## 3. Experimental Methods

### 3.1. Objects

The chest CT images of patients diagnosed with PLC by needle biopsy or surgical pathology in X Hospital from September 2016 to September 2020 were retrospectively analyzed. A total of 115 cases were included, including 83 males and 32 females, with an average age of 61.25 ± 8.48 years old (32∼80 years old) and an average lesion diameter of 2.93 ± 1.14 cm (1.00∼7.83 cm). The inclusion criteria were defined as follows: those who were diagnosed as PLC by pathological examination, those who had not received relevant treatment before CT examination, patients whose lesion was located in the west of the segmental bronchus and was a solid lesion, and patients whose lesion size was more than 10 mm. The exclusion criteria were defined as follows: patients with poor CT image quality, patients who were unable to effectively observe the lesion, and patients with other malignant tumors. Based on the results of the pathological examination, they were divided into a peripheral SCLC group and a peripheral NSCLC group (including lung adenocarcinoma and lung adenosquamous carcinoma). This study was approved by the ethics committee of X Hospital.

### 3.2. CT Scan and Image Measurement

The patients included in this study received routine CT scans. During the examination, the patient was scanned in the supine position from the lung tip to the diaphragm base. The slice thickness and spacing were 8 mm, the tube voltage was 120 kV, the tube current was 80∼120 mA, and the thin-layer reconstruction was 2 mm. The diameter of the lesion was measured on the largest axial plane. Two thoracic radiologists were required to complete the measurement on the picture archiving and communication systems (PACSS), and the average value was calculated and recorded. The CT image data of the patient's lungs obtained from the scan was transmitted to the SIEMENS workstation, and the BMP format was exported at the maximum axial level of the lesion. In addition, the window width and window level of the mediastinal window were adjusted to 350 Hu and 40 Hu, respectively.

### 3.3. Construction of LPS Algorithm Based on CNN

The Mask-RCNN model was selected for LPS in lung CT images to improve the segmentation effect of lung parenchyma. Compared with the Faster-RCNN model, the Mask-RCNN model had a more refined region of interest (ROI) alignment, which could align the selected feature region with the original image, thereby improving the accuracy of the image segmentation. Then, the full convolutional network (FCN) was applied for image segmentation [14]. The basic structure of the Mask-RCNN model is given in Figure 3.

The Mask-RCNN model applied in this study included the FPN and ResNet50 network for feature extraction in images. Compared with the conventional CNN model, the residual function was introduced into the ResNet50 network, which could effectively solve the gradient dispersion, gradient explosion, and network degradation caused by network deepening. The residual module in the network can directly transport the input value *x* to the target position through a short-circuit connection. If the mapping function of the intermediate network was set to *F*, the function output to the next layer of the network was *H*(*x*) = *F*(*x*) + *x*. The function that had to be fitted in the entire network unit could be set as *F*(*x*) = *H*(*x*) − *x*. When *F*(*x*) = 0, then *H*(*x*) = *x*, which was the identity mapping. The basic structure of the residual network ResNet50 used in this study is shown in Table 1. Except for the first group of convolutional layers, the residual blocks in the other convolutional layers were all composed of 3 convolutions. In addition, the short connection in the first residual block of each group had to be added with a convolutional layer with a convolution kernel size of 1 × 1 and batch normalization (BN) layer to achieve the feature dimension change.

The FPN was introduced to expand on the basis of the network so as to improve the feature extraction performance of the ResNet50 network. FPN covered three routes: bottom-up, top-down, and horizontal connection. The bottom-up path in the FPN was a feed-forward calculation of the ResNet50 network; the top-down path could be used for the upsampling of simple spatial resolution images to expand the feature map; the horizontal connection path could combine the features of upsampling and downsampling and match the dimension of the feature map using 1 × 1 convolutional layer. The structure of the fusion of the FPN and ResNet50 network is illustrated in Figure 4. The ResNet50 network finally generated P2 ∼ P6 feature maps corresponding to the bottom-up convolutional layers Conv2 ∼ Conv6. The underlying feature maps were mainly used for small targets, and the high-level feature maps were used for larger goals. The multiscale feature maps provided by the RPN network and the FPN network could be undertaken as the input of the ROI pooling layer, and the FCN algorithm could predict each ROI.

The ROI alignment was improved further on the basis of the ROI pooling layer of the Faster-RCNN model, which could realize the correspondence between output image pixels and input image pixels. Since the ROI pooling layer had to be quantized on the boundary of the candidate area and the boundary of different units, the obtained candidate frame deviated from the original frame to a certain degree. To make up for the shortcomings of the ROI pooling layer, it was necessary to cancel the quantization operation and use the bilinear interpolation method to replace the original nearest-neighbor interpolation method, so as to obtain the value of the image pixels and then to continuously extract the features in the image. When the image was processed, it had to calculate the target pixel position in the original image firstly:

(2) $$\begin{array}{c} \text{src}X=\text{dst}X\cdot \left(\frac{\text{src}W}{\text{dst}W}\right), \end{array}$$

(3) $$\begin{array}{c} \text{src}Y=\text{dst}Y\cdot \left(\frac{\text{src}H}{\text{dst}H}\right). \end{array}$$

In equations (2) and (3), dstX and dstY were the pixel coordinates in the recommended area, srcX and srcY were the target pixel coordinates in the original image, srcW and srcH were the width and height of the original image, and dstW and dstH were the width and height in the recommended areas.

The target pixel point was assumed to be *f* (*x* + *i*, *y* + *j*); then, the pixel value of the unit sampling point could be calculated as follows:

(4) $$\begin{array}{c} f\left(x+i,y+j\right)=\left(1-i\right)\left(1-j\right)f\left(x,y\right)+\left(1-i\right)jf\left(x,y+1\right)\\ +i\left(1-j\right)f\left(x+1,y\right)+ijf\left(x+1,y+1\right). \end{array}$$

Equation (4) was the difference between the four coordinate points in the *x* and *y* directions. Bilinear interpolation was used to calculate the pixel values of different unit sampling points, and then the maximum pooling operation was performed.

The ROI multitask loss obtained by constructing the network sampling had to be trained. The loss training methods included frame regression and target detection and classification. The calculation equation of the overall loss function of the model could be written as follows:

(5) $$\begin{array}{c} \text{Loss}={\text{Loss}}_{\text{cls}}+{\text{Loss}}_{\text{box}}+{\text{Loss}}_{\text{mask}}. \end{array}$$

The loss function Loss_mask_ of the mask in equation (5) was the average binary cross-entropy loss (ABCEL), which could be calculated as follows:

(6) $$\begin{array}{c} \text{ABCEL}\left(\text{traget},\text{output}\right)=-\left(\text{traget}\cdot \;\log\left(\text{output}\right)+\left(1-\text{traget}\right)\cdot \;\log\left(1-\text{output}\right)\right). \end{array}$$

In equation (6), *target* referred to the target value, and *output* was the actual output value of the network. For different ROIs, the classification category had to be detected firstly, and the cross-entropy error of the category branch was undertaken as the loss value for subsequent calculations. Therefore, the network needed classification to classify instead of further distinguishing the classification of pixels.

### 3.4. Extract

The CNN model is a feed-forward neural network, and it is a multilayer perceptron model constructed for recognizing two-dimensional and above images. The current CNN model includes LeNet and AlexNet models, among which the LeNet-5 model is relatively mature and the network structure is simpler. R-CNN follows the traditional idea of target detection, first extracting candidate frames, and then extracting features for each frame. Image classification and nonmaximum suppression steps detect targets, but R-CNN is low in efficiency. We use preprocessing steps such as selective search to extract potential bounding boxes as input, but R-CNN still inputs all regions to CNN, and feature extraction is still where repeated calculations appear. In the Fast-R-CNN network structure, classification, feature extraction, proposal extraction, and border regression are integrated into one network, which is conducive to the deep learning network to complete multiple tasks at the same time, and the detection speed is significantly improved. Mask-R-CNN is based on Fast-R-CNN by adding a branch to obtain a new network framework. This new mask branch is applied to the small full convolution of each ROI (Region of Interest) Neural Network, and the prediction segmentation mask is pixel-to-pixel. The Mask-R-CNN built on the basis of Fast-R-CNN is easier to train and adds a variety of flexible architecture designs. Mask-R-CNN uses bilinear interpolation to obtain the key coordinates of the small unit and performs the maximum pooling operation internally (see Figure 5).

### 3.5. Extraction of Texture Parameters in CT Images of Lung Parenchyma

The above model was adopted for LPS in lung CT images, and finally, the texture parameters in the image were extracted. Firstly, the segmented image was standardized, and the parameters in different directions (vertical, horizontal, 45°, 135°) of each ROI were calculated based on the cooccurrence matrix, and the distance *d* was adopted to represent each direction. The cooccurrence matrix parameters were to calculate the distance among the image points, and the corresponding texture parameter index was selected for subsequent extraction of texture features. Finally, 6 categories were obtained, and MaZda software was adopted to extract the texture parameters in different categories.

Histogram could show the range and frequency of pixel values in the ROI of the lesion location. The extraction parameters included contrast, correlation, sum of squares, and angular second moments.

Absolute gradient preserved the spatial information among the pixels. The extraction parameters included gradient variance, gradient kurtosis, and average absolute gradient.

The autoregressive model was to weight the intensity of adjacent pixels in the ROI of the lesion. The extraction parameters included *σ* and *θ*.

GLCM showed the number, distance, and angle of gray-level combinations in the ROI of the lesion location. The extraction parameters included mean, skewness, variance, percentile, and kurtosis.

Wavelet transformation could realize the linear transformation of the data vector. The extracted parameters included the conversion coefficient energy of different bands.

The run length matrix showed the calculation of features in different directions of the ROI. The extraction parameters included length nonuniformity, long/short run weight, and gray-scale nonuniformity.

### 3.6. CT Image Recognition and Analysis

There were many texture features in CT images of lung parenchymal calculated by MaZda software, so the dimensionality reduction of the feature was required. In this study, the Fisher coefficient method [15] was applied to reduce the dimensionality of the extracted texture features. Then, the data of texture features after dimensionality reduction were identified using principal component analysis (PCA), linear discriminant analysis (LDA), and nonlinear discriminant (NDA).

The Dice coefficient and the segmentation efficiency of the image were utilized to construct the quantitative evaluation standard of the segmentation effect of the deep learning model. Dice coefficient was a measurement function of set similarity to evaluate the similarity between samples, which could be calculated as follows:

(7) $$\begin{array}{c} \text{Dice}\left(X,Y\right)=2\times \frac{\left|X\cap Y\right|}{\left|X\right|+\left|Y\right|},\;\text{Dice}\in \left[0,1\right]. \end{array}$$

The *X* area in (7) was the resulting map of CT image segmentation by the algorithm proposed in this study; the *X* area was the effect map of manual CT image segmentation (as the gold standard). The larger the Dice coefficient value, the higher the similarity between the proposed method's segmentation effect and the gold standard [16, 17]. The extracted texture parameters were analyzed with the MLR analysis method, so as to screen the discriminative predictors of peripheral NSCLC. The receiver operating characteristic curve (ROC) curve was drawn and the area under the curve (AUC) was calculated, so as to evaluate the effectiveness of the differential diagnosis of each predictor on peripheral NSCLC. When AUC was 0.5∼0.7, it was defined as general effectiveness, AUC within 0.7∼0.9 meant medium effectiveness, and AUC within 0.9∼1.0 meant the effectiveness was high. Youden's index was applied to evaluate the specificity and sensitivity of each predictor in the differential diagnosis of peripheral NSCLC.

### 3.7. Verification of LPS Based on CNN

The hardware and software environment used for the LPS deep learning model experiment were defined as follows: Inter Xeon E5-2620 V3 central processing unit, 32G memory, Ubuntu 14.04 operating system, TensorFlow deep learning framework, and Python 3.6 third-party libraries for experimental support. The CNN model was trained and verified based on the Lung Phantom Dataset. A total of 2,500 chest CT images were selected and divided into a training set and a test set at the ratio of 4 : 1. The mask label of lung parenchyma was generated by manual labeling. The training method for constructing the CNN model was stochastic gradient descent (SGD); the number of iterations was 500; the learning rate was set to 0.0001; the weight attenuation coefficient was set to 0.0001.

### 3.8. Statistical Analysis

SPSS22.0 software was undertaken for the statistical processing of experimental data. Continuous variables were represented by mean ± standard deviation, and independent sample *t*-tests were used for difference comparison; binary variables were represented by percentage (%) data, and cards were used. The square test was adopted for difference comparison. When *p* < 0.05, the difference was considered to be statistically significant.

## 4. Experimental Results and Analysis

### 4.1. Verification of LPS Based on CNN

The effect of lung segmentation using the Mask-RCNN model is shown in Figure 6. The red box in the figure represented the area where the model was segmented.

The effects of 2D CH [18], Faster-RCNN [19], Mask-RCNN, and the improved Mask-RCNN model proposed for LPS in lung CT images were compared and analyzed, and the results are given in Figure 6. It showed that the effect of LPS by the 2D CH method was much lower in contrast to that of Faster-RCNN, Mask-RCNN, and the methods proposed. The segmentation effect of the Faster-RCNN and Mask-RCNN models was basically the same, but the detailed segmentation effect of the Mask-RCNN model was better. However, the improved Mask-RCNN model proposed showed the best effect for LPS, which could achieve the complete inclusion of lung parenchyma with a small amount of bone tissue (see Figure 7).

The efficiency of different algorithms for LPS was compared using the Dice coefficient, segmentation accuracy, and segmentation speed. Firstly, the Dice coefficients of different algorithms in LPS of the three CT images were compared.  Figure 8(a) illustrates that the Dice coefficient of the 2D CH algorithm is always the lowest, while that of the algorithm proposed is the highest. Secondly, the Dice coefficients of different algorithms for LPS of CT images on various data sets were compared and analyzed, and the results are illustrated in Figure 8(b). The average Dice coefficients of 2D CH algorithm, Faster-RCNN, Mask-RCNN, and the algorithm proposed in the validation set were 0.882, 0.953, 0.961, and 0.986, respectively. It indicated that the improved deep learning model proposed for LPS in lung CT images showed the highest similarity with the results of the gold standard segmentation.

The accuracy of LPS of lung CT images using different algorithms in the verification set was analyzed and compared, and the results are illustrated in Figure 9. It revealed that the average accuracy of LPS of the 2D CH algorithm, Faster-RCNN, Mask-RCNN, and the algorithm proposed was 88.3%, 93.5%, 94.4%, and 97.2%, respectively. It suggested that the algorithm proposed showed high accuracy in LPS.

The speed differences of LPS in lung CT images with different algorithms in the verification set were analyzed and compared. As illustrated in Figure 10, the average segmentation speeds of the 2D CH algorithm, Faster-RCNN, Mask-RCNN, and the algorithm proposed in the LPS in lung CT images were 0.289 s/sheet, 0.115 s/sheet, 0.108 s/sheet, and 0.089 s/sheet, respectively. It indicated that the image segmentation speed of deep learning algorithms had far exceeded that of traditional algorithms due to the acceleration of the graphic processing unit (GPU) [20].

As a whole, the improved deep learning model proposed showed better robustness and segmentation efficiency in LPS in lung CT images, and it could realize better fitting for the gap caused by the segmentation of blood vessels.

### 4.2. Basic Data of Patients

115 patients with PLC were included in this study, including 83 males and 32 females. They were rolled into a peripheral NSCLC group (*n* = 48) and a peripheral SCLC group (*n* = 67) according to pathological examination results. The differences in the average age, the gender ratio, and the largest diameter of the lesions of the patients were compared. As given in Table 2, there was no great difference in the average age and the largest diameter of the lesions between the two groups of patients (*p* > 0.05). The proportion of men in the SCLC group was greatly higher than that in the NSCLC group (*p* < 0.05).

### 4.3. Analysis of Texture Features of Image Segmentation Based on Deep Learning

The improved deep learning model proposed was applied to the LPS of the lung CT images of the SCLC group and the NSCLC group, and the segmentation results were compared with those of manual segmentation (gold standard). As revealed in Figure 11, the improved deep learning model could realize the LPS in lung CT images of SCLC and NSCLC patients. In contrary to the gold standard, the Dice coefficient was as high as 0.989, indicating that the segmentation results of the two methods were highly similar. Such results provided the foundation for image texture features extraction.

After dimensionality reduction of the texture features in the CT images after segmentation using the Fisher coefficients, the texture features of the images of two groups were compared. The results given in Figure 12 displayed that the SCLC group and the NSCLC group showed a visible difference in texture features of CT images after the dimensionality reduction (*p* < 0.05).

### 4.4. Evaluation on Identification Value Based on Texture Features of CT Image

The diagnostic performance of texture features parameters of each image was evaluated using the single factor analysis, and the AUC value, Youden index, sensitivity, and specificity of each image texture feature were calculated, respectively. The results in Figure 13 indicated that the AUC values of each image texture feature differential diagnosis of SCLC and NSCLC were all in the range of 0.6 to 0.7, of which *S*(4, 4)Contrast had the largest AUC. The Youden index of the differential diagnosis of texture features of each image was 0.2∼0.4, so it belonged to the general diagnostic performance as a whole. *S*(4, 0)SumVarnc had the highest sensitivity in the differential diagnosis of SCLC and NSCLC, and *S*(2, −2)SumVarnc had the highest specificity in the differential diagnosis of SCLC and NSCLC.

Then, the correlations of the above-mentioned advantages of texture features to differentially diagnose between the SCLC and NSCLC were compared using the MLR analysis. The results given in Table 3 showed that *S*(4, 4)Contrast was positively correlated with the differential diagnosis of SCLC, while *S*(4, 0)SumVarnc and *S*(2, −2)SumVarnc were negatively correlated with the differential diagnosis of SCLC.

The *S*(4, 4)Contrast in CT images of SCLC patients was higher, indicating that the correlation among pixels in CT images of SCLC patients was lower, but the contrast was higher, so the local pixel gray value difference in the image was large. This may be due to the high degree of tumor malignancy in SCLC patients, which made the difference among the textures of the image larger and reduced the uniformity [21, 22].

## 5. Conclusion

The deep learning model used for LPS in lung CT images showed good robustness and segmentation rate. The extraction and comparison of texture features of SCLC and NSCLC based on the CT image after LPS could realize the differential diagnosis of the disease. However, the effectiveness of a single CT image texture feature was analyzed in the differential diagnosis of SCLC and NSCLC only. In the follow-up, it was necessary to further explore the effectiveness of different CT image texture features in the differential diagnosis of diseases. In short, the results of this study could provide a reference for improving the efficiency of clinical differential diagnosis of SCLC and NSCLC.

## Figures and Tables

**Figure 1:** The CT images of lung nodules (a), lung adenocarcinoma (b), and lung squamous cell carcinoma (c).

**Figure 2:** The basic structure of the CNN model.

**Figure 3:** Basic structure of Mask-RCNN model.

**Figure 4:** Basic framework of ResNet50 combined with FPN algorithm.

**Figure 5:** Schematic diagram of Mask-R-CNN structure.

**Figure 6:** LPS effect based on Mask-RCNN model.

**Figure 7:** LPS effects of different segmentation algorithms.

**Figure 8:** (a) Comparison of Dice coefficients of different algorithms in LPS. (b) Comparison of Dice coefficients of different algorithms in LPS.

**Figure 9:** Comparison of the accuracy of different algorithms in LPS.

**Figure 10:** Comparison of the speed of different algorithms in LPS.

**Figure 11:** LPS results of lung CT images based on deep learning.

**Figure 12:** Comparison of texture features of CT images after dimensionality reduction. *Note.*^*∗*^indicated *p* < 0.05.

**Figure 13:** Evaluation of the effectiveness of differential diagnosis of texture features of each CT image.

**Table 1:** Basic structure and parameter settings of ResNet5.

Layer name	Output size	50-layer
Conv1	256 × 256	7 × 7, 64, stride 2
Conv2_x	128 × 128	3 × 3 max pool, stride 2
		$\left[\begin{array}{cc} 1\times 1 & 64\\ 3\times 3 & 64\\ 1\times 1 & 256 \end{array}\right]\times 3$
Conv3_x	64 × 64	$\left[\begin{array}{cc} 1\times 1 & 128\\ 3\times 3 & 128\\ 1\times 1 & 512 \end{array}\right]\times 4$
Conv4_x	32 × 32	$\left[\begin{array}{c} \begin{array}{cc} 1\times 1 & 256 \end{array}\\ \begin{array}{cc} 3\times 3 & 256 \end{array}\\ \begin{array}{cc} 1\times 1 & 1024 \end{array} \end{array}\right]\times 6$
Conv5_x	16 × 16	$\left[\begin{array}{c} \begin{array}{cc} 1\times 1 & 512 \end{array}\\ \begin{array}{cc} 3\times 3 & 512 \end{array}\\ \begin{array}{cc} 1\times 1 & 2048 \end{array} \end{array}\right]\times 3$

**Table 2:** Comparison of basic data of two groups of patients.

Item		NSCLC (*n* = 48)	SCLC (*n* = 67)	*t*/*χ*^2^ value	*p* value
Age (years old)		62.33 ± 8.49	63.18 ± 9.63	−0.528	0.789
Gender [*n* (%)]	Males	32 (66.8)	51 (76.1)	11.623	<0.001
	Females	17(35.4)	15 (22.4)		
The largest diameter (cm)		3.05 ± 1.44	3.42 ± 1.82	−0.623	0.802

**Table 3:** Correlation of texture features of CT image to identify the SCLC using MLR analysis.

Parameter	*β*	Wald	Odds ratio (OR) (95% confidential interval)	*p*
*S*(4, 4)Contrast	0.044	4.526	1.063 (0.926∼1.305)	0.031
*S*(4, 0)SumVarnc	−0.119	4.023	0.928 (0.852∼0.993)	0.043
*S*(2, −2)SumVarnc	−0.621	4.112	0.939 (0.815∼1.057)	0.039

## Data Availability

No data were used to support this study.
